# Sports Analysis and Action Optimization in Physical Education Teaching Practice Based on Internet of Things Sensor Perception

**DOI:** 10.1155/2022/7152953

**Published:** 2022-06-30

**Authors:** Mengjunguang Chen, Jingjing Jiang

**Affiliations:** Department of Physical Education, Chang'an University, Xi'an 710021, Shanxi, China

## Abstract

With the progress of the Internet of things technology in recent years, all aspects of people's lives have also been affected. More and more people are immersed in the virtual world and ignore the real activities. According to the survey, nearly 50% of people in China are in subhealth, mainly modern diseases caused by long-term inactivity. Therefore, to form a good habit of physical exercise, we must start from an early age. Starting from the physical education teaching in primary and secondary schools and from the perspective of modern scientific and technological facilities, this paper discusses the practical sports analysis and action optimization of physical education teaching based on the perception of the Internet of things. Starting from the practice of Internet of things sensor sensing in physical education teaching, we have successively determined the multisensor motion acquisition system algorithm, motion pattern recognition algorithm, and motion energy consumption algorithm, which provides modern equipment for motion analysis and motion optimization in physical education teaching practice, which breaks the current situation that traditional teachers spend a lot of time and energy for students. Combining sports mode with sports energy consumption can not only analyze sports data accurately and in real time but also optimize and predict students' sports behavior in time. We hope to supervise and urge primary and secondary school students to exercise through technical means to improve the quality of primary and secondary school students' exercise and improve people's health through physical exercise.

## 1. Introduction

The explanation and analysis of sports behavior in traditional physical education teaching is generally the model of physical education teachers' real demonstration and students' imitation. However, physical education teaching is often a teacher who teaches multiple students at the same time, lacking enough energy and comprehensive observation [1]. Even if some students spend the same time and energy on physical exercise, their behavior is not in place or standardized, resulting in ineffective exercise and even physical damage, which is extremely unfavorable to the development and growth of teenagers [2]. With the development of science and technology, more and more types of advanced equipment are constantly introduced into the teaching classroom, such as the Trinity Interactive system between students' parents and schools, large screen computers. In physical education, some schools try to use virtual reality and other types of advanced equipment for pioneering physical education [3]. The essence of virtual reality is a wearable device, which is also a research hotspot in recent years. Wearing relevant equipment during exercise can capture relevant motion data during exercise and obtain real-time data acquisition for subsequent related processing and analysis [4]. Combined with the current situation that the physical quality of primary and middle school students in China is declining year by year, we can first collect data through the physical condition or physical condition of students and then analyze the specific situation of students and formulate corresponding and reasonable training plans. This can not only make primary and secondary school students get effective exercise but also control the energy consumed by exercise, avoid excessive consumption within a reasonable range, and effectively improve students' physical quality to the greatest extent. Firstly, this paper analyzes three kinds of sports often carried out by primary and secondary school students, namely, jumping, walking, and running [5]. The Internet of things collects standard action data as the identification benchmark of subsequent actions. The acceleration speed of these three actions is very different. Therefore, the main principle of motion recognition is to judge which of the three motion modes is an action by calculating the motion acceleration of the current actual action. In addition, a series of motion data signals such as acceleration, signal amplitude, local tilt angle, and average acceleration in acceleration stage are also analyzed in this paper. Finally, the above motion recognition algorithm is combined with the Internet of things sensor technology for physical education practice analysis and motion optimization.

A good algorithm must need corresponding quantitative indexes, referring to the quantitative index of physical exercise, sports energy consumption. Therefore, we also take the energy consumed in the process of sports as the embodiment of the effect of physical exercise. At the same time, considering that different exercise modes consume different energy, different individuals perform the same exercise mode, and the energy consumption is also different due to individual differences [6]. Therefore, we propose three models to calculate the motion energy consumption under different conditions. Firstly, based on the principle of multiple regression linear model, we can roughly get the optimal value of the linear regression relationship between individual students' age, height, weight, gender, and energy consumption and then get the linear acceleration model according to different exercise forms. Based on the linear acceleration model, the relationship between acceleration and energy consumption is analyzed, and then a linear integral model is proposed. Finally, the students' motion energy consumption is estimated through the kinetic energy theorem. Because the above three models are based on different calculation principles and methods, although they are helpful to the quantitative evaluation of sports energy consumption of primary and middle school students, there are still some differences in the accuracy of the models. Therefore, this paper finally carries out a computer simulation test on the above work and analyzes the estimation results of the three models. Finally, it shows that the linear acceleration model is the most accurate for the calculation of sports energy consumption of primary and secondary school students.

Starting from the physical education teaching in primary and secondary schools and from the perspective of modern scientific and technological facilities, this paper discusses the practical sports analysis and action optimization of physical education teaching based on the sensor perception of the Internet of things. The research and innovation contributions include the following: (1) Starting from the practice of Internet of things sensor sensing in physical education teaching, we have successively determined the multisensor motion acquisition system algorithm, motion pattern recognition algorithm, and motion energy consumption algorithm, which provides modern equipment for motion analysis and motion optimization in physical education teaching practice, which breaks the current situation that traditional teachers spend a lot of time and energy for students. (2) It fully embodies the interdisciplinary characteristics; that is, it combines modern network technologies such as network communication, data acquisition computer system, and electronic sensor system, involving sports health and human movement. (3) The combination of motion mode and motion energy consumption can not only analyze the motion data accurately and in real time but also optimize and predict the motion behavior in time.

Starting from the physical education teaching in primary and secondary schools and from the perspective of modern scientific and technological facilities, this paper discusses the practical sports analysis and action optimization of physical education teaching based on the sensor perception of the Internet of things. This paper is divided into five parts. The first part expounds the explanation and analysis of sports behavior in traditional physical education teaching. At the same time, it analyzes the sports often carried out by primary and secondary school students. The second part analyzes the literature application of sports equipment sensors. From the perspective of modern scientific and technological facilities, the third part discusses the practical sports analysis and action optimization of physical education teaching based on the sensor perception of the Internet of things. The fourth part describes the model results. Compared with different models, the estimation result of linear acceleration model is the most accurate, which can be used for motion analysis and motion optimization in the practice of Internet of things sensing physical education teaching. Finally, the full text is summarized.

## 2. Related Work

In recent years, mobile devices suitable for ordinary sports lovers have been gradually listed on the market, such as Huawei smart bracelet, Nike +, Adidas MiCoach, and other mobile devices. Because these mobile devices can enable exercisers to carry and record relevant sports data during physical training, these mobile devices also belong to generalized wearable data acquisition products [7]. The emergence of these products facilitates the data collection in the training process to a certain extent. They belong to the application of sensorable technology in sports. However, such products are usually only applicable to professional sports teams or a single sports event. In the final analysis, because the algorithm of such products is relatively single, they can only collect, simulate, and analyze sports data in specific situations [8]. At the same time, the use of such products usually requires corresponding auxiliary equipment for auxiliary training, and the relevant auxiliary equipment is usually expensive [9]. For example, in the use of a common sports equipment in the market, the cost of setting up a camera alone is as high as 100000 euros. If we want to promote and use it in physical education teaching in primary and secondary schools, it is obvious that the cost exceeds the budget [10]. At the same time, this kind of equipment has a large volume and is not suitable for primary and secondary school students to wear and use at any time. To sum up, for the application of sensorable technology in sports practice and analysis in physical education teaching, there is an urgent need for a special data acquisition system to analyze action practice and wear wearable devices for action guidance and optimization.

At present, there are many research results on motion data acquisition system at home and abroad. Sport Universal Process, a French data company, has developed a sports club data analysis system especially used to analyze football match data. The essence of the system is to compare the collected data with the standard data and analyze and generate the corresponding analysis data results through the corresponding algorithm of the software. Among them, the data acquisition source of the acquisition system is mainly the high-speed cameras installed in various places in the sports field. These high-speed cameras will record the whole process of the game and generate data analysis sources [11]. German SAP data company uses match insights data analysis system to predict football solutions and analyze various game data. The system helped Germany successfully predict and win the Hercules cup at the 2014 World Cup in Brazil. The system is also equipped with supporting mobile devices and analysis applications. Through the prediction and analysis system, the football team can obtain kinematics anytime and anywhere and formulate football plans and various competition data of rival teams [12]. Nanjing University of Technology and others have also designed relevant football sports data acquisition systems. At the same time, they have cooperated with the French laboratory PROTEE to design a sports acquisition system based on a wireless sensor network [13]. Shenyang University and others designed ZigBee's motion data acquisition system and transmission module [14].

The data characteristics of different motion modes are different, so the research on motion mode recognition is also more extensive at home and abroad. By combining the relevant principles of motion mechanics and biology, Simi company of Germany has designed a motion capture and analysis system for restoring human motion posture, and the test shows that the system has high accuracy. Tian LAN and Greg Mori designed a conditional random field object recognition model based on the hiding condition principle of maximum boundary value. The design system first compares the local features with the standard data features and then integrates the local features to form a large number of global features, which are compared with the standard data features again, so as to distinguish different sports actions. The Institute of Computing Technology of the Chinese Academy of Sciences has developed a method to extract data from the moving human body under different dynamic background structures, such as running, jumping, long jump, and javelin, so as to identify different movement modes with high accuracy. Overall, the motion system is based on three-dimensional human motion simulation and video analysis and computer-aided motion recognition, extraction, and judgment [15].

The common sports index is energy consumption. The higher the flow consumption, the more effective the sports. Therefore, the data analysis system usually carries the function of identifying the amount of energy consumed. For example, American companies BodyMedia and Sense Wear wrap the arm strap of the product sent by the data collector around the exerciser's big arm, and the exerciser drives the sensor on the arm to generate relevant fluctuations through physical movement so as to obtain the exercise data during the exercise of the exerciser and analyze these data through specific algorithms and software. We can get how much energy the exerciser consumes in the exercise process so as to judge the exercise effect. Therefore, it is necessary to promote the perceptible technology in the physical education teaching of primary and middle school students so as to analyze the quality and efficiency of physical exercise. By selecting an effective sports model and reasonable energy consumption, we can objectively analyze and evaluate the overall sports process, provide scientific sports suggestions, and formulate a reasonable sports plan so as to effectively improve the physical quality of students.

## 3. Method

The key point and difficulty of sports analysis and action optimization engineering in physical education practice lie in the identification of sports mode. Only by effectively identifying the collected data can it be compared, judged, and analyzed with the standard data. The data source of this paper is that the experimenter wears sensing equipment for physical exercise and collects the experimenter's sports data through the data acquisition algorithm.

Firstly, it is necessary to determine the wearing position of the data collector. The data signals generated by different body parts are different. Therefore, the wearing position of the data collector is directly related to the authenticity and effectiveness of the collected data. Through the research on the wearing position of the existing data collector in the market, it is found that the main wearing positions are waist, wrist, upper arm, lower leg, and ankle. Through the verification of specific experimental tests, we found that when the upper limb wears the data collector, such as wrist, upper arm, and other parts, because the upper limb is an auxiliary part, different sports movements need coordinated movements of the upper limb, so there is little difference between different sports movements. Therefore, in the subsequent analysis, especially when the heat consumed by the collected action is compared and analyzed, the difference comparison cannot be made. At the same time, when the upper limb of the body moves, it usually makes a circular motion with the shoulder as the reason and the arm as the radius. Even in the in situ motion, the acceleration of the circular motion is obvious. This leads to a large amount of acceleration in the collected data, which greatly interferes with the subsequent analysis process, especially the number of motion steps.

Next, we consider wearing the data collector on the experimenter's lower limbs, such as lower legs or ankles, but the effect is not ideal. When the experimenter performs strenuous exercise, such as running or jumping, the strength and support of lower limbs are more important, so the whole lower limbs will participate, resulting in the impact of knee and ankle joints and greater friction, resulting in a large amount of irregular noise in the subsequently collected data, which cannot be separated from the real data. It is not conducive to further analysis and processing of the data collected by the data collector. At the same time, the lower leg and ankle are lower in the human body structure. During the experiment, the data collector worn on the lower leg and ankle is thrown out due to too intense leg movement, resulting in equipment damage.

This paper also considers putting the wearable device into the experimenter's pocket, but it is found that the wearable device sensor will rub a lot with the experimenter's clothes, which is not conducive to the subsequent analysis and processing of the collected data. At the same time, when wearable devices are worn on the body, it can be assumed that they are integrated and have the same acceleration. However, when the wearable device is placed in the clothing pocket, the two are separated. After the wearable device sensor is subjected to upward force, due to its different mass, it is also different from the body acceleration. Therefore, the reliability of the collected data also needs to be further reduced.

To sum up the data, the final experiment found that wearing the wearable device at the waist is the most suitable position. Firstly, the waist participates in different activities such as walking, running, and jumping, and the force and trajectory of the waist are different in different activities. Therefore, the data characteristics of the waist are the most obvious, and the data collected by the collector worn on the waist is vertical data, which changes more than the horizontal data collected by other parts. At the same time, wearing the wearable device sensor on the experimenter's waist will minimize the movement process of the experimenter. Even if it is worn for a long time, it will not affect the whole movement. Therefore, it can reflect the movement process of the experimenter to the greatest extent, and the reference value of data collection is also the greatest.

After determining the exercise mode and relevant experimental design, we will officially start the experiment. First, we randomly recruited a group of 40 primary and secondary school student volunteers, including 23 boys and 17 girls. When wearing a multisensor data collector at the waist, these experimenters carried out 5 standing long jumps, 5 5-meter run-up long jumps, 5 normal speed walks in 1 minute, 5 fast walks in 1 minute, 5 slow runs in 1 minute, and 5 fast runs in 1 minute. In order to avoid the interference of irrelevant signals, we uniformly adjusted the data sampling frequency to 50 Hz. At the same time, in order to further analyze the differences in the same exercise between different individuals, individual information such as height, weight, gender, and age was recorded at the same time. In order to ensure the accuracy of the experimental data, that is, the sports carried out by the experimenter in a good and normal state, this experiment is carried out in batches. Sufficient rest time shall be reserved between different experimental items to avoid the state after the previous exercise affecting the next exercise (see Figure 1).

After collecting the specific motion data of the experimenter through the data collector with a multisensor sensing function, due to the experimental environment and design reasons, the initially collected data inevitably contains a lot of noise. Therefore, the first step of data analysis is to clean the original data and wash away the invalid data. Firstly, we analyze the available digital signals collected by the data sensor, such as the acceleration generated by human motion and the gravity acceleration of the Earth. In addition, there is the acceleration generated by the sensor sliding due to the motion process, as well as the minor actions caused by the unavoidable environmental factors in the measurement process, such as the experimenter's own shaking or external forces such as wind. In order to avoid the influence of invalid data, that is, noise, we first improved the sensor for collecting data and put it firmly on the waist so as to reduce the noise caused by the sliding of the sensor. However, objective factors such as shaking of the experimenter or wind cannot be avoided, so we hope to clean the data by filtering method. First, assume that there is a column of ordered data:

(1) $$\begin{array}{c} a_{1},a_{2},a_{3},a_{4,}\ldots ,a_{n-1},a_{n}. \end{array}$$

If a window with a fixed length *m* (*m* is an odd number) is used for the data sequence, *m* data sequences will be taken out continuously from the original sequence at random as follows:

(2) $$\begin{array}{c} a_{i-v},\ldots ,a_{i-1},a_{i},a_{i+1},a_{i+2},\ldots ,a_{i+v}. \end{array}$$

Then, the median of the sequence is *a*_*i*_, and the median is *M*_*i*_; then, there is

(3) $$\begin{array}{c} M_{i}=\text{Med}\left\{a_{i-v},\ldots ,a_{i-1},a_{i},a_{i+v},\ldots ,a_{i+v}\right\}. \end{array}$$

Therefore, we call *M*_*i*_ the final result output value of the window crossing sequence with length *m*. In practical application, the size of *m* value directly affects the final output result. As shown in Figures 2 and 3, when the time values of the *x*-axis and *y*-axis change, the constant speed acceleration remains unchanged and is in dynamic balance. Through experiments, it is found that when the *m* value is 3, 5, and 13, the effect of data noise reduction is the best. Finally, we go to *m* = 3, process the data collected by the multisensor sensing data collector, and draw the motion acceleration relationship as follows (see Figures 2 and 3).

After data cleaning, it is necessary to analyze the cleaned data to identify the classification of motion modes as accurately as possible. Here, only three basic movements commonly used in physical education teaching in primary and secondary schools are studied, namely, walking, running, and jumping. The specific classification of each type of movement is shown in Figure 4.

Firstly, we identify jumping movement. The biggest difference between walking and running is that the first two are periodic movements. From the specific data signals, we can also see that the overall movement changes periodically. Jumping belongs to explosive movement, and the duration is short. After the experimenter took off, the acceleration value gradually decreased under the action of gravity in the ascending stage. The horizontal acceleration is 0 from the landing to the next take-off, and the vertical acceleration is about 1 g until the next take-off. Thus, the formula for calculating the take-off resultant force acceleration of the experimenter is

(4) $$\begin{array}{c} a\left(t\right)=\sqrt{a_{x}^{2}+a_{y}^{2}+a_{z}^{2}}. \end{array}$$

The left side of the equal sign represents the resultant acceleration of the experimenter, and the right side of the equation represents the motion acceleration component of the experimenter in the *X*, *Y*, and *Z* directions.

For walking and running, they have great similarity and only change greatly in step amplitude. The specific step frequency formula is as follows, but obviously, it is not accurate enough to distinguish the two movement modes only by step amplitude, so we still need other recognition conditions for reference:

(5) $$\begin{array}{c} \text{stride frequency}=\frac{\text{Total steps}}{\text{Duration of exercise}}. \end{array}$$

After determining the sports mode, in order to further analyze sports and optimize related actions in physical education teaching, we introduce the research on sports energy consumption for measurement. From the biological point of view, energy consumption is positively proportional to the product of individual mass and exercise time. The specific relationship is as follows:

(6) $$\begin{array}{c} \text{energy consumption }\left(\text{kcal}\right)=\text{weight }\left(\text{kg}\right)\times \text{exercise time }\left(\text{min}\right)\times \text{0}.179\text{.} \end{array}$$

However, the formula only considers the role of exercise time in overall exercise and does not consider the change of exercise mode on energy consumption in finishing exercise. Therefore, in the sports analysis of physical education practice, we cannot accurately understand the real sports situation of students. Therefore, we need a more accurate energy consumption calculation formula. According to the data, the linear calculation formula between accelerometer output data and energy consumption has been summarized in the experiment, which has been widely used in academia and has a high reference value. Therefore, this paper also takes it as the calculation formula of motion energy consumption. In this formula, there is a linear relationship between accelerometer output data (AO) and energy consumption. The specific formula is as follows:

(7) $$\begin{array}{c} EE=1.294\times AO+77.988. \end{array}$$

In the linear formula, *r* value and *p* value are the basis for measuring the accuracy of the model. The value of *r* is called the correlation coefficient, that is, the regression coefficient in the regression equation. The greater the absolute value of *r*, the higher the linear correlation between the independent variable and the dependent variable. We use *x*_*i*_ and *y*_*i*_(*i*=1,2,3 … *n*) to represent two variables; $\bar{x}$ and $\bar{y}$, respectively, represent the average value of the two variables, so the calculation method of *r* value is as follows:

(8) $$\begin{array}{c} r=\frac{\delta_{xy}^{2}}{\delta_{x}\delta_{y}}=\frac{\sum_{i=1}^{n}\left(x_{i}-\bar{x}\right)\left(y_{i}-\bar{y}\right)}{\sqrt{\sum_{i=1}^{n}{\left(x_{i}-\bar{x}\right)}^{2}}\sqrt{\sum_{i=1}^{n}{\left(y_{i}-\bar{y}\right)}^{2}}}. \end{array}$$

Next, we verify the accuracy of energy consumption calculation through experiments for the optimization of practical actions in physical education teaching. It is known that the normal range of body mass index of standard BMI (body mass index) is 18.5–24.99. The calculation method is as follows:

(9) $$\begin{array}{c} \text{BMI}=\frac{\text{weight }\left(\text{kg}\right)}{\text{height}{\left(\text{m}\right)}^{2}}. \end{array}$$

After determining the approximate linear relationship of the energy consumption calculation method, we began to estimate the specific calculation model through the principles of linear acceleration, linear integral, and kinetic energy theorem. The specific model is as follows:

(10) $$\begin{array}{c} \text{Motion energy consumption}=\text{a}\times \text{Kinematic acceleration}+\text{b},\\ EE_{a}\left(t\right)=a_{1}\times H\left(t\right)+b_{1}\times V\left(t\right)+c. \end{array}$$

According to relevant experimental calculations, *a*_1_ and *b*_1_ have the following linear relationship:

(11) $$\begin{array}{c} a_{1}=a_{1}\times weight\left(kg\right)+\beta_{1}\times height\left(cm\right)+\gamma_{1}\times age\left(year\right)+\delta_{1},\\ b_{1}=a_{2}\times weight\left(kg\right)+\beta_{2}\times height\left(cm\right)+\gamma_{2}\times age\left(year\right)+\delta_{2},\\ IA=IA_{x}+IA_{y}+IA_{z},\\ EE\left(t\right)=a_{2}\times IA\left(t\right)+b_{2}. \end{array}$$

To sum up, according to the principle that energy consumption is linear with individual mass and motion time and based on the principles of linear acceleration, linear integral, and kinetic energy theorem, three motion energy consumption models are proposed in this paper. The model adds the differences in motion mode and individual parameters to the original energy consumption model, which makes the calculation degree of the model more accurate.

## 4. Result Analysis and Discussion

According to the above theoretical research results, finally, we verify our theoretical results through computer simulation, that is, the performance of data acquisition system, the accuracy of motion recognition algorithm, and the accuracy of energy model consumption.

Firstly, the performance of the data acquisition system is verified. The acquisition system is tested on 8 runways of the standard 400 m playground, and the perception of the sensor is verified through the test. During the test, the sensing central machine is located above the playground facing the podium, which is generally in the middle of the whole playground. The central sensor can be used as a signal tower to communicate the transmitting end and receiving end of the collector. One person acts as a physical education teacher, which is located on one side of the central sensor and holds a signal receiving device to receive and view students' sports data in real time. Forty students wear multisensor sensing physical education teaching equipment and move randomly in the playground. After the test, the relationship between line mileage, request, and delay is shown in Figure 5. It can be seen that the delay is short and the overall acceptance is good. In order to avoid the situation that the dead corner of the playground cannot transmit data, the experiment focuses on the corners and other places. The results show that the communication between the data collector and the hardware base station is correct.

The energy consumption calculation of the traditional Meijer algorithm and the algorithm model proposed in this paper is tested. Under the condition of the same motion mode and time, it is more accurate to observe the algorithm. The specific results are shown in Figure 6.

Firstly, it can be seen from Figure 6 that the change trend of data values calculated by the three algorithms is basically the same. It can be seen that the calculation of this algorithm is basically correct, and the response is basically consistent with the energy consumption of physical exercise in physical education teaching practice. However, on the whole, the energy consumption of the three models under the same sports events is lower than that of the traditional Meijer algorithm. Through further observation, we can see that the energy consumption of the two sports modes of constant speed walking and fast running is much lower than that of other sports. According to the literature, in order to counteract the influence of gravity during walking, the human body automatically generates more acceleration in the vertical direction, resulting in the reduction of motion energy consumption in the vertical direction. To sum up, the relevant linear analysis diagram is obtained after the energy consumption of various sports indicators (Figure 7).

To sum up, the three algorithms have certain advantages. Compared with the general algorithm, the estimation result of linear acceleration model is the most accurate, which can be used for motion analysis and motion optimization in the practice of Internet of things sensing physical education teaching.

## 5. Conclusion

Starting from the practice of IoT sensor sensing in physical education teaching, this paper successively determines the multisensor motion acquisition system algorithm, motion mode recognition algorithm, and motion energy consumption algorithm to provide modern equipment for motion analysis and motion optimization in physical education teaching practice, which breaks the current situation that a traditional teacher consumes a lot of time and energy for students. At the same time, this discipline fully embodies the characteristics of interdisciplinary; that is, it combines modern network technologies such as network communication, data acquisition computer system, and electronic sensor system, and involves sports health and human movement. The combination of sports mode and sports energy consumption can not only accurately and in real time analyze sports data but also optimize and predict sports actions in time. In view of China's current attention to physical exercise and physical quality of primary and middle school students, we believe that this system has high practical value and good application products, which can be transformed into specific products in physical education teaching practice.

## Figures and Tables

**Figure 1:** Schematic diagram of wearable devices.

**Figure 2:** Acceleration-time diagram at a constant speed.

**Figure 3:** Fast run acceleration-time diagram at a constant speed.

**Figure 4:** Classification diagram of motion modes.

**Figure 5:** A large number of request environment simulation test results.

**Figure 6:** Comparison of average energy consumption calculated by different algorithms.

**Figure 7:** Schematic diagram of linear analysis of the estimated value of linear acceleration model and Meijer formula.

## Data Availability

The experimental data used to support the findings of this study are available from the corresponding author upon request.
